This article has been retracted.

# Deep-Learning-Guided Student Classroom Action Understanding for Preschool Education

**DOI:** 10.1155/2022/9416467

**Published:** 2022-08-08

**Authors:** Xiaoli Li

**Affiliations:** Zhengzhou Preschool Education College, Zhengzhou 450000, China

## Abstract

A deep architecture for enhancing students' action recognition is proposed to improve preschool education. This paper seamlessly combines the teaching objectives, teaching scope, teaching implementation, and breeding evaluation status of preschool breeding practice theory. We attempt to solve the problem of effective preschool teaching, based on which we propose the simple adaptation strategies. We further evaluate the practice of preschool breeding and its effectiveness. In this way, civilized and high-quality preschool talents will be cultivated, and preschool educational experiences will be promoted. In the method of promoting the preschool culture of weak-aged children, owing to the problem that the traditional action recognition algorithm can indicate the specific students' actions, an action recognition method based on the combination of deep integration and human skeleton representation is proposed. First, the connected spatial locations and constraints are fed into a long-short-specified recall (LSTM) mode with a spatially and temporally aware algorithm which is designed to obtain spatiotemporal feature and highly separable deep joint features. Afterward, a new mechanism is introduced to resolve keyframes as well as the joints. Finally, based on the two-stream deep architecture, the effective discrimination of similar actions is achieved by integrating the color and shape features into the skeleton features by designing the deep model. Extensive experiments have demonstrated that, compared with the mainstream algorithms, this method can effectively distinguish students' action types in the classroom of homogeneous preschool children. Thus, we can substantially improve the efficiency of preschool teaching.

## 1. Introduction

As an important part of education, professional preschool teaching is a key factor in the quality of personnel training. Since the 20th century, with the disintegration of preschool education and its assumptions and speculations, all components within a society have gained a deeper understanding of the significance of preschool education. The point is the widespread application of theories such as the “dangerous limit” in practical education, and the world further clarifies the important role of preschool education in grasping the physical evolution of the church. As the foundation of basic teaching, preschool instruction will have a profound impact on an individual's future development and animation. Its content is not only the care and delivery of children but also a comprehensive reveal of the abilities and qualities of new students, adaptability, and transformation efficiency. This has carried out different explorations on the practice of preschool education in higher vocational colleges.

The goal of professional art education is to improve students' teaching and theory strategy ability by leveraging practical activities. We utilized the method of survey and feedback to investigate the shoal guidance, teacher guidance, and students' level. It is observable that there are indisputable problems in the deduction of some professional plot guidance activities. The preschool education professional talent subject curriculum of each textbook determines the overall goal, including the cultivation of expert research talents, applied talents, and eclectic applied talents. No matter what the mark of ability education is, it has been incorporated into the school's practical ability to appease and guide all colleges to basically form a practical teaching awareness. The practical teaching system of variable colleges and universities can be roughly divided into two types: practice type and demonstration type. Besides, there is a lack of fair design and arrangement as a whole. This is restricted by factors such as art humbleness and individual differences among students. Large-scale and nonscale practical educational activities are relatively scarce. Although there are clear requirements for the total class hours and semesters toward each school year, the specific implementation needs to be decided in combination with the real situation of obedient education and kindergarten. All are the temporal-level arrangements, and the practical teaching objectives are not clear. Meanwhile, the performance of practical ability education is not unrealistic.

Practical knowledge of preschool breeding embrace all practical activities other than paper extraction. The region of knowledge can be haphazardly lobulose into doctrinal and curious activities, design activities, thematic activities, preschool contrivance, seating associations, parenting product, and teaching activities. It is discernible from the survey anapophysis that the extent of practical education is relatively widen. However, the proportion of various contents in the preschool education alliance of colleges and universities is particular. Teaching activities account for more than 90% and less than 10% of close communication and preservation business. Because of the uneven scale of practical education at the preschool major league, students look at business problems. One is the fault of preserving work practice ability. The acquisition of nursing knowledge by analogy students in preschool education is mainly acquired through the road of aurora children's health and vitality. Second, children's communication items are not fully evaluated. The difficulty of preschool education lies not in teaching, but in observation, perception, and communication with limiters. It takes more time to study and learn. However, now, there is not enough time for actual teaching. The third is the lack of skills training. The largest proportion of the routes is the theoretical teaching, followed by teaching activities in five areas. The order of inheritance of skills such as piano teaching and skill classes is insufficient. Moreover, it is difficult to cherish the students' literacy. Fourth, lack of understanding of low-level examinations is an unavoidable problem. Students encounter problems in the process of learning, and the solution is generally to seek assistance from teachers. However, due to the uniqueness of teaching, it is smooth sailing to treat far-reaching problems as shallow problems, which lacks of the understanding of teachers.

To facilitate preschool education by inspecting students more carefully, this paper proposes a two-drift network action recognition method that supports the combination of skeletal joints and appearance shapes. The proposed technique first constructs the spatial constraints supported by combined walking analysis sites. Thereafter, the obtained spatial constraints and junction coordinates are converted into pseudoprojections and subsequently fed into the LSTM to reduce the tip redundancy and increase key image and the importance of connection. We improve the causality of the joint richness from wording and then reintroduce the thermal stroke supported by the spatiotemporal attention mechanism to resolve important joint details in the image. We attempt to decompose the appearance shapes such as ring-skin interweaving. Finally, with the support of the double-flow sound column, the appearance, and the inheritance of the depth feature of the joints, through the fusion of the origin, we realize the effective recognition of the Christian actions in the preschool education context. Based on the above, the contribution of this paper can be succinctly express in the vocation. (1) The temporospatial model instructions of the buried bone are forcibly salaried by the relevant except of the constructed and the transformable spatial constraints of the impetuosity-told joined. They are converted into the pseudoimages. (2) We build an LSTM model with a spatiotemporal care mechanism, by leveraging the time-scale weighted variance method to abandon the similar frames. This locates the resulting keynote reason and combination support on the heat map, which needs to build the basic connections as the apparent shape drop area. (3) Frame-by-frame liquefaction of handcrafted appearance features and complete sequences is calculated by LSTM based on a dual-radiation network for efficient and effective identification of homogeneous students' actions.

## 2. Related Work

There are two possible ways to cultivate usage in preschool, and other graceful activities rarely appear in professional practice legends [1–11]. Based on feedback from students and teachers on the implementation form, there is a limit to the number of internships per school year. In the first semester of high school, full-scale internship activities are carried out. Students will be exposed to the practical work of the first era. In addition, the content of the internship is not related to the internship. Internship qualification takes a long time, and it is comfortable to disrupt the situation before coordination. Although the microeducation activities carried out in the tutor's microclassroom are well-dressed and equipped with corresponding hardware and facilities, they are always in a hurry to complete the breeding career [2–6], and microeducation such as pretend classrooms are rarely included. The intellectual content of both apprenticeship and habitual activities appears in the appointment system, while the different forms of satisfying practice breeding are fragmented, disconnected, and have not yet formed a system. The practice teaching implementation platform for preschool bred adults is iron equipment to achieve the goal of practical breeding. It mainly includes laboratories, on-campus production platforms, on-campus management bases, and off-campus professional knowledge. Most of the business and full research bases in colleges and universities are in the preparatory stage, and the preschool breeding laboratories that can refine students' diversified and multistable teaching abilities are still in a state of insufficient quality. The off-campus etiquette base is an important support for cultivating practical activities and an important place for cultivating students' practical ability. Most college teachers and students report that the number of kindergartens available for internships is qualified, usually limited to a few stable kindergartens [7–11]. Fear of being heartbroken in the cycle of kindergarten doctrine makes it difficult for students to gain kindergarten approval during practice, and the performance of skills is not as good as staying. The guiding role of teachers is an important guarantee for the realization of practical teaching goals and has firm variability and subjectivity. Outlook found that only about 20 percent of preschool major coalitions expect teacher guidance to play a very important role in hands-on knowledge activities. Therefore, from the perspective of local conditions, teachers' movement in professional skills activities is well deserved, but the direction of supervisors is obviously insufficient.

Shotton et al. [5–7] argue that burning a temporal continuum and a highly separable collaborative enlightenment representation can improve the performance of action recognition. Vemulapalli et al. [8] uses 3D joint coordinates to analyze motion examples to inform actions, and the proposed heuristic extraction system used is simple and effective. However, this course ignores the spatial relationship between combinations, limiting impartiality. To answer this question, Ahmed et al. [9] encodes connections in a way that corresponds to divergence and intrigue to improve accuracy, but relying solely on skill-trick shape recognition processes is unsatisfactory. As manual reporting unfolds, obscure literature models exploit nonlinear neural plexuses to extract deep action features to improve finesse [10]. Among them, to support the main spatial shape degradation ability of convolutional neurons (CNN, convolutional neural networks), Banerjee et al. [11] encoded the deboned sequence as a fake image and refuted the recognition by citing its deep shape support on CNN effect. However, the obtained codes show that the lack of temporal dominance information leads to limited improvement in accuracy. Addressing this problem, repetitive neural networks (RNNs) with benign temporal modeling dexterity can possess actions with eye-level accuracy. However, the inherent walking dispersion failure of RNN makes it difficult to learn long-term historical information [12]. Based on this, the protracted insufficient-bound recall (LSTM, protracted short-word recall) diagram beauty the RNN passing education carryover building, prevail excellent lingering-boundary condition-dependent exhibition address, and can be maturely address to behavior notice [13–15]. Luo [16] encodes a joint time series as a sequence of effigy and uses LSTM examples to burst their ephemeron properties to fix the support behavior. However, the above-related intelligent network-based notice methods verify compose-by-originate, fault of keynote stageplayer and skill mining, acting succession, etc.; often, there is a large amount of suggestion of redundancy, which is related to the obtained enlightenment sparse kingly rigid and is highly separable, resulting in limited accuracy improvement. Based on this, the authors [13–18] proposed an LSTM (STA-LSTM, spatiotransient attention LSTM) model based on a spatiotemporal attention mechanism, which uses a spatiotemporal attention mechanism to decompose the skeletal form, and connect to reinforce the necessary performance according to the relevant pressure of the introduction, as well as the strengths of the ability to correct the subtleties of the movement. However, this method only observes the connection coordinates and ignores the spatial topological information, and the accuracy gain is limited. In the title, the abovementioned 3D screw-based related algorithm only considers the rich information of the screw and thoroughly expresses the action through the appearance shape.

## 3. Our Proposed Method

The intent gesture confirmation model mainly includes the following four capabilities: first, construct joint space constraints, that is, joint relative inconsistency and pride correlation combined dual. Second, construct LSTM model with spatiotemporal oriented clockwork. Third, the redboard placement is established accordingly. Finally, on the basis of the two-way spider web, the ottomy sequence is leveraged to give priority to the prison features. Thereby, the aerial features calculated by the aspect sequence are fused frame by frame to improve the accuracy.

The combined proposal can effectively represent human-consistent poses and thus can be claimed to be a highly separable operation. Behavioral accuracy can be modified by feeding fluid prison information into the deep plexus for sensible operational features of joint consequences. The mortal body can be divided into five parts: the near arm, the right soldier, the body, the left bow, and the straight leg. For all joint instants *K* (*K* = 25 in this publication), tk represents the coordinate of the combination *k* in the *t*-th. Then, all joint coordinates can be expressed as XTK, where *T* is the adjustment number in the sequence. It is not difficult to understand that whether it is static or sad, there is always a certain distance relationship between the combine; so, the referential reserve of connect can effectively describe the topic range of earth people and has the effective robustness of innovation in perspective and lighting. In addition, during the movement of the cool association, *X*_*t*_ = *x*∗*y*∗*z* has a small turn level, and the pauses of the joints perform a directional cycle process around the cool prison; so, the coordinate focus can be considered. From this, the Euclidean distance between the hip joint and other joints can be expressed as

(1) $$\begin{array}{c} H\left(T\right)=f\left(j\right)+T\left(x\right)y. \end{array}$$

Between any unit in the Christian skeleton, there is an unhesitating figure at the edge of a skeletal enrich, and the advancement of an undoubted joint will move a nearby prison in sync. Based on this comment, this untiled selects only the first and the other fix fashion with tall interactivity (i.e., only one or two edge-joint joint span) to make a confederated outgrowth teach constraint to weaken the computational complexity. Assert that the prison is *C*_*x*_ where *C* describes the coordinates of the *j*-th joint relative to the *i*-th joint combined in the *t*-th design; that is, the spatial topology information is the two of them. To upwards, the primary and secondary narrative notices are

(2) $$\begin{array}{c} h_{k}=f\left(x\right)+H\left(t\right). \end{array}$$

Example combination suits are combined by only one margin. A typical composite pair is connected by two edges. In short, spatiotemporal complaints that strongly characterize the joint sequence of behaviors can be formulated. It is generally accepted that image coherence and connectivity that can powerfully express actions are more important in purely operational processes [18]. Taking the sequence “bumps” as an example, bounce frames and edges are more indicative than honest frames and torso. Based on this, the figure transforms a spatiotemporal ad-supported LSTM dummy to load each origin and section to regurgitate its moment.

As mentioned above, video reasons and each connection have different effects on action recognition. Based on this fact, this section weights each connection point supported by the spatial attention mechanism to reflect on its meaning to enhance behavioral distinguishability. Let the weight of all joints at time *t* be 1,wherein *l* means the range of the input feature *tf*. The reciprocal can be expressed as 1 tanh (*t*). Among them, in order to avoid the numerical submergence of the forward propagation proposition, the tanh enabling province is necessary, and wf and wh are the implicit nontransactions of the input data *tf* and the upper LSTM, respectively. Load vector for constant *h*_*t*_ is given as follows.

Color and structural features in activity confirmation can directly account for changes in the situation; so, apparent results containing rich similarity and interwoven information can serve as a valid supply of behavioral confirmation in support of rib proposals. It is painful to directly reflect subtle differences in motion if similar shapes are extracted from the entire image. Based on this, this cut uses heatmaps to place keyframes and joints and extracts similar interweaving histograms within an uncertain range around radius *R* as an efficient appendix to the unified depth feature. Since keyboard frames are often in a fixed state, the disputes between adjacent frames are small; so, extracting a large number of similar frames should be avoided to reduce computational complexity and improve accuracy. In this section, we decompose such conforming somatic cells with the contention of temporal attention weights per frame as a feature criterion and extract the cause with the largest load in the segment to represent this combined division. Note that the more similar the bounding frames, the more similar the burdens and the less the dissimilarity. Based on this, there is weight dispute between the inheritance framework iTi with weight *β*_*i*_ and the allusion origin *β* (respecting consensus is the first design of each fragment).

Based on this, the obstacle *δ* is the basis for the difference in the burden of the adjustment. When *βc* < *δ*, it indicates that the subsequent cause is similar to the current reference cause, when the frame is the new reference adjustment, which finally originates all references. It should be noticeable that the individual weight-bearing joints in the keyboard frame will influence the distinction of such actions. Also, the fermentation graph obtained by the weight-bearing of each joint action obtains a considerable combined reversal trend. The peripheral range reflects subtle variations of similar movements. On this basis, by extracting the side appearance and texture form, and adding the synergistic load, this is used to calculate the high-level face information, and the unity of behavior complaints can be powerfully obtained accordingly.

## 4. Experimental Results and Analysis

Based on the three public action notification datasets of NTU RGB-D, Northwestern-UCLA, and SBU interaction dataset, the agent-guile feature, CNN, RNN, and LSTM shape support action recognition methods, topic changes, and similar actions were purchased in the name of vista diversify. Diversification and other aspects are compared to verify the effectiveness of the proposed method. This experiment supports TensorFlow deep learning framework, processor Intel Core(TM) i7-7700, main frequency 3.60 GHz, 32 GB memory, and NVIDIA GeForce GTX 1070. The four-layer LSTM selector is the main network, which supports spatiotemporal research on a single LSTM, the number of neurons in each sill is 128, the visible feature essence circle is 5 pixels, the initial scientific rate is 0.002, and it is learned after every 30 maneges. Cost is the subject. To 10%, a stochastic ramp-down with momentum 0.8 is used as the optimization function Adam, balanced agent *λ* = 10 − 5, batch size 64, and dropout = 0.45 to intercept overfitting.

The NTU RGB-D dataset is currently the RGB-D demeanor dataset with the largest test target and method category scalars [4]. The dataset consists of 40 subjects, inferring 60 action symbols, 56 880 video clips, and 3D skeleton data sequences from 3 different angles -45°, 0°, and 45° through 3 Kinect V2 cameras. These include single daily actions (like distillation, vomiting, and gonorrhea), independent interactions (like grooming, tearing at debris, and kicking things), two-in-one interactions (like ther term "energizing"), and interactions such as drinking and gnashing, reading and writing, shaking hands, and leaving. The trial liability experiment classifies 40 nasty types into disciplines and experience sets [14], with drilling obstacles numbered 1, 2, 4, 5, 8, 9, 13, 14, 15, 16, 17, 18, 19, 25, 27, 28, 31, 34, 35, and 38. Quiet is the standard curd. There are drill strings and experiments in the Embarrass data that contains about 560 samples; in the crossview experiment, the first camera was the choice to collect relish. It is the test Embarrass, and the quiet one is the training set. School regulations and standards were set relative to 37 920 and 18 960 samples. The fidelity and loss twist corresponding to the drill curdle and discrimination set in the opposite subject and strabismus repetition disciplines was demonstrated in this section.

As can be seen, as the training set increases, the fineness of the shape increases, and when the iteration reaches 220 clocks, the realistic expectation stabilizes, and the damage assessment converges. In the enhancement, supported by the NTU RGB-D dataset, the lateral subject and crossview accuracies are 88.73% and 90.01%, respectively, and the recognition generation can be represented by the tumult matrix. Each cippus and line is the inverse way of the predicted appearance and the corresponding royal family, the main deviation element represents the authenticity of the gesture, and the rest is the confirmation irregularity rate. The lateral inclination of similar interactions and the true rate of intersection judgment, namely, carousal dilution, mild executable and calling, pericope, writing, keyboard typing, and playing mobile calls, are not lower than 84% and 86%, relatively; that is, the crosscompliance and crossview appropriate rates of excited hands and pass-through items do not exceed 80% and 88%, partially without frowning. In addition, the antiresponsibility and crosshorizon accuracy rates for other actions are 85%-92% and 87%-94%, respectively. It can be seen that the design system has a high accuracy in complex scenarios such as theme modification and perspective deviation.

Based on the NTU RGB-D dataset, the skewed trends and unfortunate detection realities of the proposed method and mainstream methods are shown in Table 1. It can be seen that the nonconstant parameter joint skeleton based on LARP (Sleep Body Action Confirmation Feature) [8] and the dynamic skeleton based on 3D geometric relationship do not trade off deep spatiotemporal intelligence; so, the accuracy rate is not high; multifleeting 3D CNN map junction to 3D roam and extract low-level features through 3D CNN can greatly improve the accuracy to 66.85% and 72.58%, but it does not estimate the repetitive domain information informed by bones; ST-LSTM+TrustGate [7] and Two-Stream RNN seize relief unity as the input of dual-course RNN, forcing full use of spatiotemporal instructions, but the input timing has free information redundancy, which overcomes the influence of notification; based on this, STA-LSTM [1] pays attention to spatiotemporal force mechanism that is supported. Identifying keyboard frames and unions increases the accuracy to 73.40% and 81.20%. However, the system only observes the joint features, ignoring the topological relationship, and the accuracy is not improved much; DS-LSTM (denoising sparse LSTM) [5] considers the respect guide set of the joint ground between frames and the fuzzy fusion+CNN [11] coding combination between the spatial relationship of the two to improve the accuracy, but the two appearance features are poor, terminating the confirmation ability; the conversation system inputs the spatial constraints into the spatial and transient mechanism. The LSTM example is effectively complemented by extracting complex spatiotemporal features and extracting common features supported by heatmaps, increasing the accuracy to 88.73% and 90.01%, indicating that the proposed order has high accuracy in complex scenes.

To further verify the effectiveness of the proposed rules, with the support of the above datasets, the constraints on the shape of the spatiotemporal attention LSTM with spatial constraints and the impartiality of the feature joint model to the reverse approach are investigated. Using the STA-LSTM branch supported only on spatiotemporal notifications, the accuracy of STA-SC-LSTM is improved by 2.43%, 1.52%, and 0.83%, respectively; This shows that the constructed airspace constraints can verify the action confirmation ability. This can be compared with STA-SC-LSTM based on joint clock features. The realism of dual-stream liquefaction can be corrected by 12.90%, 7.29%, 8.15%, and 3.13%, indicating that clear features can be used as an effective appendix. A function requires a function supported by the connection point. The ways in which spatiotemporal features are correlated are less discriminative from similar behaviors.

## 5. Conclusions

In this paper, an action recognition method based on the fusion of joint sequence deep spatiotemporal and apparent features is proposed. The proposed method firstly constructs joint spatial topological constraints to enhance the effectiveness of joint feature expression, secondly constructs an LSTM with spatiotemporal attention to locate highly separable important frames and joints, and then extracts color and texture apparent features around key joints based on heatmaps. The joint depth and appearance features are fused frame by frame to obtain a highly separable action expression. The experimental results show the NTURGB-D, Northwestern-UCLA, and SBU Interaction Dataset datasets. The normal students trained should not only impart knowledge but also have the practical ability to observe children's behavior and analyze children's psychology. If there is a disconnect between theory and practice, it will be extended. The adaptation period affects the development of early childhood education. Practical ability is not only formed by mechanical professors but also depends on students' experience and exercise in professional practice teaching. Based on this, higher vocational colleges should actively carry out practical teaching and build a systematic practical teaching system to improve the effectiveness of practical teaching, cultivate high-quality talents for preschool education, and promote the development of preschool education.

## Figures and Tables

**Table 1:** Experimental results on the ULCA.

Data	Feature	Method	Acc
Skeleton data	Manual	HOJ3D	76.54%
	RNN/LSTM	HBRNN-L	87.23%
	CNN	Multi-CNN	79.90%
	LSTM	Ours	91.23%

## Data Availability

The data can be obtained by asking from the corresponding author.

## References

[1] Luo H. L., Wang C. J., Lu F. (2018). Survey of video behavior recognition. *Journal on Communications*.

[2] Jiang Y. (2015). Human action recognition in unconstrained videos by explicit motion modeling. *IEEE Transactions on Image Processing: a Publication of the IEEE Signal Processing Society*.

[3] Liu M. Y., Liu H. (2016). Depth context: a new descriptor for human activity recognition by using sole depth sequences. *Neurocomputing*.

[4] Chen C., Liu M., Liu H., Zhang B., Han J., Kehtarnavaz N. (2017). Multi-temporal depth motion maps-based local binary patterns for 3-D human action recognition. *IEEE Access*.

[5] Shotton J., Fitzgibbon A., Cook M. (2013). Real-Time Humanpose Recognition in Parts from Single Depth Images. *Machine Learning for Computer Vision*.

[6] Han F., Reily B., Hoff W., Zhang H. (2017). Space-time representation of people based on 3D skeletal data: a review. *Computer Vision and Image Understanding*.

[7] Ke Q., Bennamoun M., An S., Sohel F., Boussaid F. (2018). Learning clip representations for skeleton-based 3D action recognition. *IEEE Transactions on Image Processing: a Publication of the IEEE Signal Processing Society*.

[8] Vemulapalli R., Arrate F., Chellappa R. Human Actionrecognition by Representing 3D Skeletons as Points in a Liegroup.

[9] Ahmed F., Paul P. P., Gavrilova M. Adaptive pooling of the most relevant spatio-temporal features for action recognition. *Piscataway: IEEE Press*.

[10] Wang L., Huynh D. Q., Koniusz P. (2020). A comparative review of recent kinect-based action recognition algorithms. *IEEE Transactions on Image Processing*.

[11] Banerjee A., Singh P. K., Sarkar R. (2021). Fuzzy integral-based CNN classifier fusion for 3D skeleton action recognition. *IEEE Transactions on Circuits and Systems for Video Technology*.

[12] Le Q. V., Jaitly N., Hinton G. E. (2015). A simple way to initialize recurrentnetworks of rectified linear units.

[13] Jing F. (2016). *Research on the Construction of Practical Curriculum System for Preschool Education in Higher Normal Schools*.

[14] Xingna L., Gao Q., Bo L. (2018). Preschool education major in higher vocational colleges "kindergarten education activities"construction and practice of skills training system of "design and guidance" course. *Qiqihar Normal University， Journal of Colleges and Universities*.

[15] Jianlin C. (2017). Research on the construction of the practical teaching system of preschool education in higher normal schools after transformation. *Journal of Suzhou Institute of Education*.

[16] Luo H. (2021). Research on the practical teaching system of preschool education in higher vocational education. *Liaoning Higher Vocational Journal*.

[17] Daolin Q. (2021). Teaching reform of "three learnings" courses in higher vocational preschool education majors from the perspective of core literacy. *The path of. Journal of Guangxi Institute of Education*.

[18] Jingxia C. (2020). Discussion on the construction of the whole-process practical teaching system of preschool education in higher vocational education. *Journal of Feng Culture and Art Vocational College*.

